# Curative Effect Observation and Prognosis Analysis of Video-Assisted Thoracic Surgery and Thoracotomy in Patients with Hemopneumothorax

This article has been retracted.

**DOI:** 10.1155/2021/3937420

**Published:** 2021-10-16

**Authors:** Honglei Zhang, Qian Yang, Tao Liu, Yu Liu

**Affiliations:** ^1^Second Department of Thoracic Surgery, Xingtai People's Hospital, Xingtai, Hebei 054000, China; ^2^Second Department of Thoracic Surgery, East District, Handan Central Hospital, Handan, Hebei 056008, China; ^3^Department of Emergency Surgery, The First Hospital of Yongnian District, Handan, Hebei 057150, China

## Abstract

Currently, the incidence of hemopneumothorax is high in China, and with the continuous improvement of modern medical standards, video-assisted thoracoscopic surgery (VATS) has gradually become the main method of clinical treatment of hemopneumothorax. The aim of this study was to investigate the minimally invasive mechanism and the clinical value of television thoracoscopy in the diagnosis and treatment of traumatic hemopneumothorax and to provide a relevant theoretical basis for the superiority of television thoracoscopy. In this study, total of 98 patients with traumatic hemopneumothorax admitted to three hospitals from January 2017 to December 2019 were selected and divided into 49 cases each in the thoracotomy group and VATS group according to the differences of the surgical method. The surgical situation such as operation time, intraoperative bleeding, and incision length, postoperative recovery such as duration of painkiller use, chest tube retention time, volume of drainage, and hospital stay, levels of C-reactive protein (CRP), tumor necrosis factor-*α* (TNF-*α*), interleukin-6 (IL-6), and other inflammatory factors at different times after admission to hospital, postoperative complications such as pulmonary infection, enveloped effusion, incisional infection, and pressureulcers, and recurrence rate at 12-month follow-up were used as the evaluation indexes to analyze the effect of different surgical treatment modalities in patients with hemopneumothorax and the impact on patient prognosis. The results showed that the operative time, intraoperative bleeding, duration of painkiller use, chest tube retention time, and hospital stay were shorter in the VATS group than in the thoracotomy group. The length of the surgical incision, volume of drainage, and inflammatory factor levels at different postoperative periods were lower in the VATS group than in the thoracotomy group. The incidence of postoperative complications was lower in both groups, and the difference was not statistically significant. The follow-up results showed that there were no recurrent cases in both groups 12 months after discharge. This indicates that VATS is an effective treatment option for hemopneumothorax, which can achieve the same exploration and treatment effect as thoracotomy, and has the advantages of less trauma, less bleeding, shorter operation time, and faster postoperative recovery compared with thoracotomy. The prognosis of patients treated by VTAS is good, which provides a new treatment route for patients who cannot tolerate thoracotomy and are poorly tolerated.

## 1. Introduction

Hemopneumothorax is the phenomenon of accumulation of excess gas and blood in the thoracic cavity due to trauma, spontaneous, medical malpractice, and other causes of injury to the chest tissues and organs, among which hemopneumothorax due to trauma is the most common [1]. Traumatic hemopneumothorax mostly occurs from injuries to the pleura, lungs, or bronchi caused by chest trauma such as severe chest crush injuries, rib fractures, and sharp forceps [2]. Some data [3] show that the probability of hemopneumothorax in chest trauma in China can be as high as 60%–70%, especially in recent years, sharp knife stab wounds have increased significantly, and traumatic hemopneumothorax has become a common chest trauma in general hospitals. Due to the presence of tension in pneumothorax and chest haemorrhage, patients with traumatic hemopneumothorax usually have a high mortality rate, but timely and effective treatment can save patients' lives to a great extent [4]. In the past, the treatment of traumatic hemopneumothorax was mainly based on traditional thoracotomy and closed-chest drainage, which have certain efficacy but also have more drawbacks [5, 6]. With the increasing maturity of minimally invasive clinical techniques, VATS has gradually become the direction of thoracic surgery, which has expanded the scope of thoracoscopic use because of its advantages of no aggravation of the original injury, more rapid surgery, more reliable hemostasis, faster postoperative recovery, less pain, and shorter hospital stay [7, 8]. Currently, VATS has achieved good clinical results in the treatment of thoracic trauma and has been applied to the diagnosis and treatment of a variety of thoracic traumas [9].

In this study, 98 consecutive patients with traumatic hemopneumothorax operated during the same period were selected, and different groups of patients were treated with thoracotomy and VATS respectively. Surgical situation such as operation time, intraoperative bleeding, and incision length, postoperative recovery such as duration of painkiller use, chest tube retention time, volume of drainage, and hospital stay, postoperative inflammatory factor levels at different times, postoperative complications, and recurrence rate at 12-month follow-up were used as evaluation indexes to analyse and compare the differences in trauma to the body between the two surgical procedures in order to further explore the feasibility of VATS in the treatment of hemopneumothorax.

## 2. Information and Methods

### 2.1. General Information

98 patients with traumatic hemopneumothorax treated in three hospitals from January 2017 to December 2019 were collected. Among them, 62 males and 36 females were aged from 30 to 59 years, with an average of (37.29 ± 5.43) years, and the course of disease was 1 to 6 days, with an average of (3.70 ± 1.56) days. 98 patients with traumatic hemopneumothorax were divided into 49 cases each in the thoracotomy group and VATS group according to the surgical approach. The basic data such as gender, age, nature of injury, comorbidity, and site of bleeding were compared between the two groups, and the differences were not statistically significant (*P* > 0.05, Table 1) and were comparable.

### 2.2. Inclusion Criteria

1. Patients with chest trauma with moderate or above pleural effusion confirmed by CT, with or without pneumothorax, or drainage of >1000 ml by puncture for 1 time and continuous observation of drainage of >200 ml/h per hour for 3 h or more
2. Meeting the indications for surgery
3. Patients or patients' families were informed of the treatment plan used and had signed the consent form

### 2.3. Exclusion Criteria

1. Patients with low tolerance to surgery
2. Patients with hemodynamic instability or combined cardiac macrovascular injury or abdominal injury
3. Patients with psychiatric disorders and history of cancer
4. Patients with combined immune diseases, infectious diseases, and coagulation disorders
5. Combination of severe primary diseases of vital organs

### 2.4. Treatment Methods

#### 2.4.1. VATS Group

The instruments used for the procedure were the Storz video-assisted thoracoscopy series, and bipolar electrocoagulation knife (Sabre 2400) was used for the dissection procedure. Patients were operated under general anesthesia with double-lumen intubation, in the healthy-side position with the upper arm of the affected side hoisted, and the healthy-side lung ventilation mode was used during the procedure. The incision location was the 6th or 7th intercostal space in the midaxillary line with an incision length of approximately 1 cm to 1.5 cm, and all blood clots and blood accumulation at the incision site were cleaned out after insertion of the thoracoscope [10]. The surgeon observed the patient's injury in the chest cavity through the video-assisted thoracoscopy and made two other incisions for the operation according to the exploration. The incision locations were the 3rd intercostal space in the anterior axillary line and the 5th intercostal space in the posterior axillary line, the length of the incision was also 1–1.5 cm, and the three holes should be made in an inverted triangle as much as possible when making the incision. The site of bleeding was found and then treated differently depending on the specific situation [11–13]. For bleeding in intercostal blood vessels, arteries, etc., it should be sutured or electrocoagulated to stop the bleeding in time. For patients with diaphragm injury and bleeding, titanium clips or sutures should be used for treatment. For patients with penetrating diaphragmatic injuries, it was necessary to enlarge the rupture of the diaphragm to observe whether the organs were damaged and suture the rupture of the diaphragm with a 10-gauge suture. In patients with lung lacerations, the lung was closed with continuous sutures with 3–0 Prolene sutures if the injury is superficial, and the severely injured lung tissue was removed using an endoscopic cutting closure if the lung laceration is large or penetrating. In case of pericardial laceration, the pericardial laceration needed to be enlarged appropriately to view the surface of the heart, while giving fenestration drainage and finally cleaning the chest cavity using warm saline. Drainage was routinely placed at the end of surgery and removed after chest X-ray showed complete pulmonary recruitment. During the postoperative hospitalization, appropriate pain management was given, and the dose of pain medication was determined according to the actual condition of the patient.

#### 2.4.2. Thoracotomy Group

Patients were operated under general anesthesia with dual-chamber intubation or single-chamber intubation. We take the healthy-side lying position and lift the upper arm of the affected side and choose standard lateral incision or anterior external incision according to the position of the wound. A direct incision was made through the 5th or 6th intercostal space to reach the chest cavity, and then, the patient's chest cavity was explored and the accumulated blood and clots were cleaned up; the follow-up treatment principles are the same as the VATS group.

### 2.5. Observation Indicators

1. We observed and recorded the operative conditions such as operative time, intraoperative bleeding, and incision length, postoperative recovery such as the time of analgesic drug use, chest tube retention, drainage, and hospital stay, the levels of inflammatory factors such as CRP, TNF-*α*, and IL-6 at different times after surgery, and postoperative complications such as pulmonary infection, enveloped effusion, incisional infection, and pressureulcers. The patients were followed up by telephone or outpatient clinic once every 1 month within 6 months after discharge to observe the recovery and recurrence of patients, and once every 3 months after 6 months, with a total follow-up period of 12 months, and the recurrence rate of patients in both groups was recorded.
2. Laboratory tests: the levels of serum CRP, TNF-*α*, and IL-6 were measured before surgery (T0), on day 1 (T1), day 3 (T2), day 5 (T3), and day 7 (T4) after surgery, respectively. 3∼5 ml of patients' fasting blood in the morning was collected and centrifuged at 3000r/min for 30 min at room temperature and plasma specimens were separated, and serum CRP, TNF-*α*, and IL-6 levels were measured by ELISA. The serum CRP ELISA kit, serum TNF-*α* ELISA kit, and serum IL-6 ELISA kit were purchased from Shanghai ExCell Biology Inc., and the relevant operations were carried out in strict accordance with the kit instructions.

### 2.6. Statistical Analysis Methods

The data of this study were organized and entered using EXCEL software, and the differences between the two groups were analyzed using SPSS22.0 statistical analysis software, and graphs were made using Prism8.0. The statistical data were expressed as (case, %) using the chi-square test, and the measurement data were expressed as mean ± standard deviation (mean ± SD) using the *t*-test. Data comparison was considered statistically different at *P* < 0.05.

## 3. Results

### 3.1. Comparison of Surgical Conditions between the Two Groups

The intraoperative conditions of the two groups were counted. The mean operative time, intraoperative bleeding, and incision length were (127.56 ± 32.26) minutes, (402.28 ± 143.46) mL, and (19.79 ± 2.57) cm in the thoracotomy group. In the VATS group, they were (84.39 ± 37.51) minutes, (209.53 ± 89.78) mL, and (8.22 ± 1.43) cm, respectively. The results of the comparison showed that the operative time, intraoperative bleeding, and incision length were lower in the VATS group than in the thoracotomy group, and the differences were statistically significant (*P* < 0.05, Figures 1(a)–1(c).

### 3.2. Comparison of Relevant Indexes between the Two Groups after Surgery

The postoperative conditions of the two groups were observed. The duration of analgesic use, drainage, chest tube retention, and hospital stay were (8.53 ± 1.24) days, (467.58 ± 91.43) mL, (5.34 ± 1.40) days, and (14.89 ± 2.67) days in the open-chest group and (5.26 ± 0.87) days, (307.13 ± 70.22) mL, (3.17 ± 1.21) days, and (10.36 ± 2.41) days in the VATS group, respectively. Comparing these indicators, the results of statistical analysis showed that the duration of painkiller use, chest tube retention time, volume of drainage, and hospital stay were shorter in the VATS group than in the thoracotomy group, and the drainage flow was lower than that in the open-chest group, with statistically significant differences (*P* < 0.05, Figures 2(a)–2(d)).

### 3.3. Comparison of Serum Inflammatory Factor Levels between the Two Groups at Different times

There was no statistically significant difference in the preoperative serum CRP, TNF-*α*, and IL-6 levels between the two groups (*P* > 0.05). Serum CRP, TNF-*α*, and IL-6 levels in all patients increased significantly and reached a peak on postoperative day 1 and then gradually decreased. In dynamic monitoring at 1, 3, 5, and 7 days postoperatively, serum CRP, TNF-*α*, and IL-6 levels were lower in the VATS group than in the thoracotomy group, with statistically significant differences (*P* < 0.05, Figures 3(a)–3(c)).

### 3.4. Comparison of Postoperative Complications and Recurrence between the Two Groups

Postoperative complications in both groups included pulmonary infection, encapsulated effusion, incisional infection, and pressure sores, all of which improved significantly after timely and effective management. In the thoracotomy group, there were 3 cases of pulmonary infection, 3 cases of enveloped effusion, 4 cases of incisional infection, and 3 cases of pressureulcers, with a total incidence of 26.53% (13/49). In the VATS group, there were 2 cases of pulmonary infection, 3 cases of enveloped effusion, 2 cases of incisional infection, and 1 case of pressureulcers, with a total incidence of 16.33% (8/49). The incidence of postoperative complications was lower in the VATS group than in the thoracotomy group, but the difference was not statistically significant (*P* > 0.05, Figure 4). The follow-up results showed that there were no recurrent cases in either group 12 months after discharge.

## 4. Discussion

Hemopneumothorax is one of the common complications of chest trauma, and some studies have reported that more than 60% of chest trauma patients have different degrees of hemopneumothorax, resulting in hypotension, pallor, shortness of breath, chest tightness, and other symptoms, which can cause aggravation such as hemorrhage in the chest cavity if not treated in time and may even cause death of patients in serious cases [14, 15]. In the past, the treatment of traumatic hemopneumothorax was usually carried out by means of debridement sutures and closed-chest drainage, and the decision of whether to open the chest for exploration was made according to the size of chest drainage, which was not conducive to the judgment of the patient's condition at an early stage and delayed the timing of treatment [16]. Thoracotomy allows exploration of the patient's chest cavity and timely and effective treatment, which has been a better tool for hemopneumothorax management in the past [17]. At this stage, however, the trauma caused by thoracotomy and the occurrence of postoperative complications make it difficult for the physician to decide whether to perform thoracotomy to staunch bleeding [18]. With the continuous development of minimally invasive surgical techniques, VATS provides a new way to treat traumatic hemopneumothorax, which has a clear field of view and fine instruments, and its lens and operator can enter the chest cavity and explore the damage to the patient's intrathoracic organs at a faster speed, providing good prerequisites for appropriate treatment measures for the patient in the first place [19, 20].

The results of this study showed that the operative time, intraoperative bleeding, time to analgesic medication, time to chest tube retention, and hospital stay were shorter in the VATS group than those in the thoracotomy group; the length of surgical incision and drainage were lower than those in the thoracotomy group. This result suggests that VATS treatment causes less trauma and less pain to the patient's body, which is more conducive to rapid postoperative recovery. Moreover, VATS can directly observe the situation in the patient's chest cavity and reduce the blindness in diagnosis, which can avoid misdiagnosis and delay due to diagnostic errors to a certain extent and facilitate clinicians to develop more active and effective treatment [21]. Through years of practice and the clinical characteristics of traumatic hemopneumothorax, we believe that, in patients with traumatic chest injury, especially hemopneumothorax caused by sharp penetration, VATS is recommended in all cases except for those with small wounds, mild clinical symptoms, stable vital signs, and a small amount of hemopneumothorax as confirmed by CT chest and other imaging studies.

As surgery produces unavoidable trauma to the patient's organism, the inflammatory response that occurs at the wound site causes the patient to show transient higher expression levels of inflammatory factors in the postoperative period. Inflammatory factors such as CRP, TNF-*α*, and IL-6 are commonly used clinically to assess the degree of inflammatory response [22]. CRP is a common acute phase protein, which is generally low in the blood and rises sharply when the body is exposed to infection, trauma, or surgical trauma [23]. IL-6 is a multipotent cytokine with a wide range of functions, which is rapidly produced during acute inflammatory responses such as internal and external injuries, surgical procedures, and infections, and is a major indicator of early inflammation in the organism [24]. TNF-*α* is a pleiotropic proinflammatory factor involved in the development of local inflammatory responses, and it is also often used as a clinical indicator to detect the degree of inflammatory response in the organism [25]. By measuring the levels of CRP, TNF-*α*, and IL-6 in patients with traumatic hemopneumothorax at different times, we found that both groups of patients exhibited elevated levels of the abovementioned inflammatory factors at 1 day postoperatively, which suggested that acute inflammatory reactions occurred in patients after surgery. However, the levels of inflammatory factors in the VATS group were significantly lower than those in the open-chest group at different postoperative periods, which showed that VATS was less traumatic than traditional thoracotomy surgery, highlighting the advantages of minimally invasive surgery. Postoperative complication rates were lower in patients in the VATS group than in the open-chest group, but the difference was not statistically significant, which may be related to the small sample size included in this study, but the results were equally able to show that VATS treatment has a high safety profile. There was no recurrence at 12-month postoperative follow-up, indicating that patients treated by different surgical modalities had a good prognosis.

## 5. Conclusions

VATD surgery has significant advantages over traditional thoracotomy in the diagnosis and treatment of traumatic hemopneumothorax and offers a new treatment pathway for patients, while ensuring efficacy and fewer postoperative complications.

## Figures and Tables

**Figure 1:** Comparison of surgical conditions between the two groups. (a) The average surgery time. (b) Mean intraoperative bleeding. (c) Average incision length. Compared with the thoracotomy group, ^*∗*^*P* < 0.05.

**Figure 2:** Comparison of relevant indexes between the two groups after surgery. (a) Average duration of analgesic use. (b) Average chest tube indwelling time. (c) Average volume of drainage. (d) Average hospital stay. Compared with the thoracotomy group, ^*∗*^*P* < 0.05.

**Figure 3:** Comparison of serum inflammatory factor levels between the two groups at different times. (a) Average CRP level. (b) Average TNF-*α* level. (c) Average IL-6 level. Compared with the thoracotomy group, ^*∗*^*P* < 0.05.

**Figure 4:** Comparison of postoperative complications and recurrence between the two groups.

**Table 1:** Comparison of baseline data between the two groups.

Data		Thoracotomy group (*n* = 49)	VATS group (*n* = 49)	*χ* ^2^ or *t* value	*P* value
Age (years, mean ± SD)		37.47 ± 5.76	37.08 ± 5.21	0.352	0.726

Disease duration (days, mean ± SD)		3.63 ± 1.58	3.74 ± 1.53	0.350	0.727

Gender (case, %)	Male	30 (61.22)	32 (65.31)	0.176	0.675
	Female	19 (38.78)	17 (34.69)		

Nature of injury (case, %)	Open injury	42 (85.71)	43 (87.76)	0.089	0.766
	Closed injury	7 (14.29)	6 (12.24)		

Complications (case, %)	Lung contusion	27 (55.10)	29 (59.18)	0.167	0.683
	Rib fractures	21 (42.86)	18 (36.73)	0.383	0.536
	Other	1 (2.04)	2 (4.08)	0.344	0.558

Bleeding site (case, %)	Left	36 (73.47)	34 (69.39)	0.200	0.655
	Right	13 (26.53)	15 (30.61)		

## Data Availability

The data used during the current study are available from the corresponding author on reasonable request.
